# Ppm1b Negatively Regulates 3-Bromopyruvate Induced Necroptosis in Breast Cancer Cells

This article has been retracted.

**DOI:** 10.3389/fonc.2020.555546

**Published:** 2021-01-14

**Authors:** Yiming Sun, Qiong Pan, Linyan Ma, Chao Chen, Surong Zhao, Hao Liu

**Affiliations:** ^1^ Department of Pharmacy, The First Affiliated Hospital of Bengbu Medical College, Bengbu, China; ^2^ School of Pharmacy, Bengbu Medical College, Bengbu, China

**Keywords:** breast cancer cells, protein phosphatase 1b, necroptosis, dephosphorylation, 3-bromopyruvate

## Abstract

Up to 30% of breast cancer mortality is caused by cancer relapse despite primary clinical treatments due to distant metastases. Further research focusing on breast cancer mechanisms are needed for deeper understanding of disease prognosis. 3-bromopyruvate (3-BP), a glycolysis inhibitor, has been studied as one of the antitumor agents in recent years. In this report, we want to investigate the form of cell death induced by 3-BP and demonstrate the inhibitory effect of 3-BP on breast cancer cell proliferation and its mechanism *in vivo and in vitro*. We found that 3-BP could inhibit MDA-MB-231 and MCF-7 breast cancer cell proliferation, through energy metabolism inhibition. Further, necroptosis characters in MDA-MB-231 cells after 3-BP treatment were observed, which could be negatively regulated through Ppm1b by dephosphorylation of RIP3. In addition, 3-BP treatment in an MDA-MB-231 cell-transplanted mouse model showed a significant antitumor effect, which correlated with necroptosis-related protein Ppm1b. The findings demonstrate the potential for 3-BP in the treatment of breast cancer, providing impetus for further clinical studies.

## Introduction

Breast cancer is one of the dominant types of cancers, which affects public health, especially in women (1, 2). Previous studies suggest that, up to 30% of the patients die due to distant metastatic formation (3), and patients with metastatic breast cancer survive no more than 1 year (4). Hence, various strategies need to be explored to understand mechanisms involved in breast cancer and to provide better clinical treatment.

3-BP is a small reactive molecule formed by bromination of pyruvate, which is one of the widely studied compounds due to its antitumor properties (5). A glycolysis inhibitor, 3-BP can inhibit cancer cell proliferation through energy metabolism interruption (6), primarily through inhibition of the glycolytic enzymes and those related with mitochondrial function, including hexokinase II (HK II) (7), pyruvate dehydrogenase (PDH) (6), glyceraldehyde-3-phosphate dehydrogenase (GAPDH), lactate dehydrogenase (LDH), and by altering adenosine triphosphate (ATP) levels (8). We had previously demonstrated the antitumor properties of 3-BP both *in vitro and in vivo* which was achieved through energy metabolism alterations, in colon cancer cells SW480 and HT29 treated with 3-BP, by inducing their necroptosis and apoptosis (9). Further, 3-BP enhanced antitumor activity of daunorubicin (DNR) in breast cancer cells through monocarboxylate transporter 1 (MCT-1) (10), suggesting that 3-BP could be an effective therapeutic target for breast cancer treatment.

Necroptosis is a type of programmed cell death with morphological characteristics of necrosis, associated with the kinase activity of caspase 8, receptor−interacting serine/threonine kinase 1 (RIP1), and receptor-interacting serine/threonine kinase 3 (RIP3) (11). When caspase 8 is inhibited or is deficient, RIP1 combines with RIP3 to form the RIP1/RIP3 complex *via* the-terminal RIP1 homotypic interaction motif (RHIM) domain, which initiates necroptosis (12). This confirms that the RIP1/RIP3 complex forms the core of necrosome, however, understanding of molecular regulation of necroptosis remains limited. A recent study showed that protein phosphatase 1b (Ppm1b) selectively suppresses necroptosis through dephosphorylation of RIP3, which then prevents the recruitment of mixed lineage kinase domain-like protein (MLKL) on the necrosome (13).

In this study, we report the cell death forms induced by 3-BP, we found that 3-BP, a glycolysis inhibitor can induce cell death in breast cancer cells, MDA-MB-231 and MCF-7, respectively, especially in MDA-MB-231 cells by regulating Ppm1b and necroptosis, which are crucial for our understanding of breast cancer cell death signaling network.

## Materials and Methods

### Cell Lines and Cell Culture

Breast cancer cells MDA-MB-231 and MCF-7 were obtained from the cell research institute of the Chinese Academy of Sciences (Shanghai, China). Both cells were cultured in Dulbecco’s Modified Eagle’s Medium (DMEM) (Gibco, USA), and supplemented with 10% fetal bovine serum (FBS), 80 U/ml penicillin and 100 U/ml streptomycin. Cells were grown in an atmosphere of 5% CO_2_ at 37°C.

### 3-(4, 5-Dimethylthiazol-2-Yl)-2, 5-Diphenyltetrazolium Bromide Assay

3-(4, 5-Dimethylthiazol-2-yl)-2, 5-diphenyltetrazolium bromide (MTT) (Beyotime Institute of Biotechnology, Wuhan) was used to determine cell viability. MDA-MB-231 and MCF-7 cells (5000 cells/well) were seeded onto 96-well plate and then treated with different concentrations of 3-BP (0, 20, 40, 80, 160, 320 μmol·l^-1^) (Sigma-Aldrich, USA) when cells were attached completely. MTT solution (15 μl; 5 mg/ml in phosphate-buffered saline) were added into 96-well plate respectively at the 3-BP treatment of 24, 48, and 72 h. After 4 h, the solution was replaced with 150 μl dimethylsulfoxide (DMSO) (Beyotime Institute of Biotechnology, Wuhan) and 30 min later, cell viability was determined at a wavelength of 490 nm by a microplate reader (Synergy, BioTek, USA).

### Flow Cytometry

Prior to 3-BP treatment, MDA-MB-231 and MCF-7 cells (1.2×10^5^ cells/well) were seeded onto 12-well plate and then treated with 3-BP (0, 80, 160, 320 μmol·l^-1^) for 24 h when cells were attached completely, then stained by PI solutions for 2 h, then detected by Accuri C6 flow cytometry (BD Biosciences, State of New Jersey, USA). To further analyze cell death, PI staining was used to detect cell death. Annexin-V FITC/PI staining (Nanjing keygen biotech, Nanjing) was used to detect the amounts of apoptosis cells by the method just described according to the manufacturer’s instructions.

### Nuclear Staining

DAPI nuclear staining (Beyotime Institute of Biotechnology, Wuhan) assay was performed to examine the effects of 3-BP on cancer cell apoptosis. MDA-MB-231 and MCF-7 cells were seeded onto 6-well plates (2×10^5^ cells/well). Cells were fixed with immunostaining setting for 30 min at 4°C after 3-BP treatment for 24 h, washed twice with PBS and then incubated with DAPI solution for 30 min at 4°C in the dark. The plates were then washed with PBS to remove the excess DAPI solution and the cell nuclei were observed under a laser confocal scanning microscope (LCSM, Olympus 1x71).

### Determination of ATP Level

ATP levels were measured using a luminescence-based ATP Assay Kit (Beyotime Institute of Biotechnology, Wuhan). In this assay, luciferase catalyzes the production of a fluorescent signal from oxygen, ATP, and luciferin, and the fluorescence intensity is proportional to the amount of ATP. Cells (1.2×10^5^ cells/well) were seeded onto 12-well plate and incubated with various concentrations of 3-BP for 5 h at 37°C. After 24 h, all cells were collected and homogenized in radio immunoprecipitation assay (RIPA) lysis buffer for 10 min on ice, and then centrifuged at 12000 *g*/min for 5 min at 4°C. Next, 100 μl nucleotide-releasing buffer and 1 μl ATP-monitoring enzyme were added to each well of a 96-well plate, and 30 μl cell suspension was transferred into each well. The plate was then incubated at 25°C for 60 s, and the fluorescence was measured using a Luminoskan luminometer (Thermo Scientific, Atlanta, GA, USA).

### Determination of Lactate Dehydrogenase Level

Cells (6000 cells/well) were seeded onto a 96-well cell culture plate so that the cell density does not exceed 80%–90%. Aspirate the culture medium and wash it once with PBS. Replace with fresh culture medium, and divide each culture well into the background blank control wells, control wells and drug wells, and incubated at 37°C. Then add the LDH release reagent provided by the kit, mix by pipetting several times. After reaching the predetermined time, the cell culture plate was centrifuged with a multi-well plate centrifuge at 400 g for 5 min. Take 120 μl of supernatant from each well, add Insert into the corresponding wells of a new 96-well plate, and then LDL levels were measured (Beyotime Institute of Biotechnology, Wuhan).

### Small Interfering RNA Transfection

The Human Ppm1b siRNA (Gene Pharma, Shanghai, China) was transiently transfected into MDA-MB-231 cells in a 6-well plate with Lipofectamine 2000 reagent (Invitrogen, USA) according to the manufacturer’s protocol. After 48 h of transfection, the cells were collected for immunoblot analysis. The sequences of siRNA used for experiments of human Ppm1b siRNA were as follows: Negative control sense, 5’- UUCUCCGAACGUGUCACG UTT-3 and antisense, 5’-ACGUGACACGUUCGGAGAATT-3’; Positive control sense, 5’-UGACCUCAACUACAUGGUUTT-3’ and antisense, 5’-AACCAUGUAGUUGAGGUCATT-3’; Ppm1b-homo-1728 sense, GCUGAC UAGUUACAGGCUATT and antisense, UAGCCUGUAACUAGUCAGCTT; Ppm1b-homo-1129 sense, CCAACA GAACAACUUGUUUTT and antisense, AAACAAGUUGUUCUGUUGGTT; Ppm1b-homo-1458 sense, GGAGAAGUCUGGCGAGGATT and antisense UUCCU CGCCAGACUUCUCCTT.

### Western Blotting

MDA-MB-231 and MCF-7 cells were lysed in RIPA lysis buffer on ice for 30 min, then centrifuged (12000 g/min; 30 min) at 4°C. A bicinchoninic acid (BCA) assay was used to detected protein concentrations. Equal amounts of total protein were separated by sodium dodecyl sulfate-polyacrylamide gel electrophoresis (SDS-PAGE) and transferred to polyvinylidene fluoride (PVDF) membranes (millipore, USA), and then incubated with primary antibodies overnight at 4°C after the membranes were blocked (5% skim milk in PBS with 0.1% Tween 20) for 4 h. The next day, the membranes were imaged with gel imaging equipment (Bio-Rad, USA) after the membranes were incubated with secondary antibodies for 2 h. β-actin was used as a loading control. The following antibodies were used: Bcl-2 and Bax (Cell Signaling technology, USA); anti-RIP1, anti-RIP3, and p-RIP3 (Santa Cruz Biotechnology, USA); TNF-α (Abcam, USA); Caspase 3 (Enzo, USA); Ppm1b (BETHYL, USA); anti-β-actin (Biosharp, China) All reagents were dissolved according to the manufacturer’s instructions.

### Live Cell Imaging System

MDA-MB-231 and MCF-7 cells (1.2×10^5^ cells/well) were seeded onto 12-well plate and then treated with 3-BP (0, 160 μmol·l^-1^) combined with Annexin-V (5 μmol·l^-1^), PI (5 μmol·l^-1^), and DAPI (5 μg/ml) solution when cells were attached completely. The plate was placed under a live cell workstation microscope for 24 h persistent observation, then the final video was analyzed by The Live cell imaging system (ZEISS, Germany).

### Evaluation of Cell Death Form by Electron Microscopy

MDA-MB-231 and MCF-7 cells (1.2×10^5^ cells/well) were seeded onto 12-well plate and then treated with 3-BP (0, 160 μmol·l^-1^), then collected cells, washed and fixed with 2% paraformaldehyde and 3% glutaraldehyde in 0.1 M PBS (pH 7.4) at 4°C overnight. Then, the cells were post-fixed with 1% osmium tetroxide for 1.5 h, washed once by PBS and treated with 3% aqueous uranyl acetone for 1 h before being dehydrated with a graded series of ethanol and acetone and embedded in Araldite. Thin sections were cut using a Reichert ultramicrotome (Leica, Germany), post-stained with 0.3% lead citrate, and examined by TEM (Olympus JEOL, Peabody, MA, USA).

### Xenograft Model

This study was performed according to guidelines approved by the Bengbu Medical College Institutional Animal Care and Use Committee (No. 2017003). Female nude mice (BALB/c) aged 4–5 weeks and weighted 18–20 g were used to perform the antitumor effect *in vivo*, which were obtained by Shanghai slac laboratory animal. Mice were grafted subcutaneously in the right flank with MDA-MB-231 cells resuspended in 0.2 ml PBS (10^7^ cells/ml), then randomized into negative control (PBS), 3-BP (8 mg/kg), Nec-1 (40 mmol·l^-1^) (Sigma-Aldrich, USA), 3-BP combined with Nec-1 (8 mg/kg; 40 mmol·l^-1^), DNR positive control (5 mg/kg) (Sigma-Aldrich, USA) when tumor volume reached approximately 100 mm^3^ (n=6 per group). Tumors were measured with caliper and volume was calculated by the formula: 0.5×a×b^2^, where a and b were tumor length and width. Tumors were stored in 4% formalin solution, embedded in paraffin, and stained with hematoxylin and eosin (H&E) and used for immunohistochemistry.

### Statistical Analysis

The experimental results were analyzed by SPSS 21.0 software. Data are expressed as the mean ± SD of three experiments. The differences between the groups were compared by one-way ANOVA. Mean differences were evaluated by t-test analysis of variance. *P* < 0.05 was considered statistically significant.

## Results

### Cell Proliferation Were Inhibited by 3-Bromopyruvate in Breast Cancer Cells

To identify the cell proliferation inhibition effect of 3-BP in breast cancer cells, we examined the cell viability in MDA-MB-231 and MCF-7 cells, both cell viability is inhibited by 3-BP (**Figures 1A, B**). For further confirmation, we also determined that 3-BP induced apoptosis in both cell lines (**Figure 1C**), as 3-BP could reduce cellular ATP level (**Figure 1D**). And increase cellular LDH level in MDA-MB-231 cells, while no significant change of LDH level in MCF-7 cells (**Figure 1E**).

**Figure 1:** Inhibition effect of proliferation in breast cancer cells by 3-BP. **(A)** Breast cancer cells MDA-MB-231 and MCF-7 cells were treated with 3-BP (0, 20, 40, 80, 160, 320 μmol·l^-1^) for 24, 48, and 72 h. Cell viability was measured using the MTT assay. **(B)** The cell death rate in MDA-MB-231 and MCF-7 cells induced by 3-BP for 24 h. **(C)** Cell apoptosis induced by 3-BP in MDA-MB-231 and MCF-7 cells for 24h. **(D, E)**. Reduction in ATP production and LDH level by 3-BP treatment, cells were cultured with 3-BP (0, 40, 80, 160, 320 μmol·l^-1^). Cellular levels of ATP were measured after 5 h. LDH level was measured after 24 h. *P < 0.05, **P < 0.01.

### 3-Bromopyruvate Induced Breast Cancer Cells Apoptosis and Necroptosis

To identify the apoptosis induced by 3-BP in breast cancer cells, we examined the apoptosis-related proteins, up-regulated expression of Bax and down-regulated expression of Bcl-2 mean that breast cancer cells could be induced apoptosis by 3BP (**Figures 2A, B**). Especially, cell viability in MDA-MB-231 increased in 3-BP combined with the Nec-1 group than the 3-BP group, which means that 3-BP may induce breast cancer cells MDA-MB-231 necroptosis (**Figure 2C**).

**Figure 2:** Cellular apoptosis and necroptosis induced by 3-BP in breast cancer cells. **(A, B)**. Apoptosis-related proteins were detected after cells were treated with 3-BP for 24 h, and were analyzed by western blotting. β-actin served as the loading control. **(C)**. Cells were treated with 3-BP or 3-BP combined with Nec-1 for 24 h, and cell viability was determined using MTT assay. **(D)** Cells were treated with 3-BP (0, 160 μmol·l^-1^) for 24 h and then prepared for Electron Microscopy analysis. Scale bar: 2 μm; **(E)** Cells were treated with 3-BP (0, 160 μmol·l^-1^), and observed under a live-cell workstation microscope for 24 h persistent observation. **(F)**. Cells were treated with 3-BP (0, 80, 160, 320 μmol·l^-1^) for 24 h, subjected to DAPI staining and then visualized under a fluorescence microscope. *P < 0.05, **P < 0.01.

Results shown that plasma membranes of MDA-MB-231 cells was disrupted after incubated with 3-BP for 24 h, and cell fragments are visible, resulting in the release of cell contents and swollen nuclei (N). MCF-7 cells treated with 3-BP demonstrates apoptotic cell death characteristics, with typical apoptotic bodies and the number of apoptotic nuclei had significantly increased in both the cell lines treated with 3-BP. On the other hand, necrotic symptoms such as swelling of the cell body and rupture of the cell membranes could be observed in MDA-MB-231 cells treated with 3-BP (**Figure 2D**).

Live-cell observation also shown that necroptosis characteristics, including plasma membranes, were disrupted in MDA-MB-231 cells after incubation with 3-BP (**Figure 2E**, **Supplementary Video 1**). Cell membrane valgus Annexin V/FITC combines with it and emits green light in cells early apoptosis, cell membrane swells and ruptures, and PI enters the cells, making it emits red fluorescence when 3-BP stimulates MDA-MB-231 cells for 240 min, and MCF-7 cells are mainly dominated by cell body shrinkage, which proves that 3-BP induced necrotic apoptosis in MDA-MB-231 cells and 3-BP induced MCF-7 apoptosis (**Figure 2E**, **Supplementary Video 2**). Further, cell permeability of MCF-7 cells increased, which is consistent with the Nec-1 results (**Figure 2C**). DAPI staining shows nuclear damage in both the cells indicating apoptosis (**Figure 2F**).

These observations reinforce the notion that 3-BP induces apoptosis in breast cancer cells MDA-MB-231 and MCF-7, while necroptosis in MDA-MB-231 cells.

### Ppm1b Negatively Induced Necroptosis by Dephosphorylation-Receptor−Interacting Serine/Threonine Kinase 3

Previous researches have shown that Ppm1b negatively induced necroptosis by dephosphorylation-RIP3 (13). To identify the function of Ppm1b in necroptosis in different cancer lines, we tested the expression of Ppm1b in normal human colon cell line FHC, HT29 and SW480, and breast cancer cells MDA-MB-231, MCF-7, and MDA-MB-453, we found that 3-BP could inhibit the expression of Ppm1b in MDA-MB-231 cells, with up-regulated expression of TNF-α and p-RIP 3, while no significant change in expression of RIP3 in MCF-7 cells (**Figures 3A, B**). The expression of Caspase 3 shown that apoptosis induced by 3-BP in MCF-7 cells. Knockdown of Ppm1b in MDA-MB-231 cells shown that Ppm1b could negatively up-regulate the expression of p-RIP3 (**Figures 3C, D**).

**Figure 3:** Ppm1b negatively induced necroptosis by dephosphorylation-RIP3. **(A, B)** MDA-MB-231 cells were treated with 3-BP (0, 160 μmol·l^-1^), Protein expression of Ppm1b, TNF-α, RIP3, p-RIP3, Caspase 3, and β-actin were analyzed by western blotting. β-actin served as the loading control. **(C, D)** MDA-MB-231 cells were transfected with siRNA against Ppm1b, then Ppm1b and p-RIP3 were analyzed by western blotting. β-actin served as the loading control. *P < 0.05; **P < 0.01.

These observations reinforce the notion that 3-BP induced breast cancer cells MDA-MB-231 necroptosis and Ppm1b negatively regulated 3BP-induced necroptosis through dephosphorylating RIP3.

### Anti-Tumor Effect of 3-Bromopyruvate in Breast Cancer Xenograft Model

To examine the anti-tumor effect of 3-BP in breast cancer *in vivo*, we performed a mice model using the breast cancer cell lines MDA-MB-231 stimulated with 3-BP. 3-BP could reduce tumor volume and tumor weight (**Figures 4A–C**) compared with the control group, with no significant liver damage (**Figure 4E**). H&E staining results shown that 3-BP induced tissue damage with no significant liver and kidney damage, while 3-BP combined with Nec-1 could reduce the tissue damage (**Figure 4F**).

**Figure 4:** Anti-tumor effect of 3-BP *in vivo*. **(A, B)** Comparison of the transplanted tumor volume. **(C, D)** Bodyweight and tumor weight were monitored every 4 days and calculated using the formula: length x width^2^/2. **(E)** ALT and AST level in mice blood after 3-BP treatment. **(F)** H&E staining *in vivo*. *P < 0.05, **P < 0.01.

In the tissue, the expression of Ppm1b in the 3-BP group was down-regulated by 3-BP than the control group, which could be released by 3-BP combined with Nec-1, and no significant change in expression of RIP3 (**Figure 5A**). Electric Microscope results shown that 3-BP induced disruption of cellular membrane and release of cell contents (**Figure 5B**), shown that 3-BP induced necroptosis *in vivo*, which consistent with the results *in vitro* (**Figure 2D**).

**Figure 5:** Necroptosis induced by 3BP *in vivo*. **(A)** Expression of Ppm1b and RIP3 in tumor tissue were detected by immunohistochemistry. then visualized under a fluorescence microscope. **(B)** Mice were treated 3-BP for 24 h, and necroptosis in tumor tissue were detected by Electron Microscopy analysis.

## Discussion

Cellular necroptosis is a necrotic programmed cell death modality pathway in a caspase-independent fashion and is mainly mediated by RIP1 (14) and RIP3 (15). Accumulating evidence suggests that necroptosis serves a double-edged sword to the development of the cancer process, performs an anti-tumor effect in cancer, or plays a tumor-promoting role in cancer development (16, 17). While much remains to be fully elucidated about the mechanism and regulation of necroptosis, given that necroptosis can be potential for developing a novel approach in cancer therapies (18).

Ppm1b is another type 2C protein phosphatase (PP2C) family member in human, which controls numerous cellular functions by dephosphorylation of serine and threonine residues, and binds to the phosphorylated TBK1 and acts as a TBK1 phosphatase (19). On the other hand, Ppm1b was found in associating with the IKKβ/NF-κB pathway (20), overexpression of Ppm1b can block the activation of the IKKβ/NF-κB pathway induced by TNF-α treatment (21). Furthermore, Ppm1b plays an important role in the progression of cells.

Published data have provided evidence of the interaction between necroptosis and protein Ppm1b *in vivo* and *in vitro* (13). It was shown that gene deletion of Ppm1b regulates necroptosis through dephosphorylating RIP3. Our data support this conclusion in breast cancer cell lines. In this investigation, we found that the anti-tumor effect of glycolysis inhibitor 3-BP in breast cancer cells, which regulated apoptosis in MCF-7 cells and MDA-MB-231 cells, with novel cell proliferation inhibition effect. These observations reinforce the notion that 3-BP suppresses breast cancer cells proliferation. We also found that 3-BP induced necroptosis in MDA-MB-231 cells, which was consistent with our previous research (22). Especially, dephosphorylating RIP3 induced by the Ppm1b depletion pathway seems to be the more dominant mechanism of 3-BP induced necroptosis in MDA-MB-231 cells (**Figures 2C, D**). Although the interaction of Ppm1b with p-RIP3 in MDA-MB-231 cells (**Figures 4A–C**) explains the role of Ppm1b in preventing necroptosis in breast cancer cells and *in vivo* (**Figures 5A, B**), the mechanism of Ppm1b during necroptosis is still unclear.

In view of the data presented here and in previous reports, it will be valuable to test the function of Ppm1b in necroptosis in the future. Taken together, the present study has identified Ppm1b as a novel phosphatase of RIP3 and provides new insight into the molecular mechanism in breast cancer cell necroptosis.

## Conclusion

In conclusion, our results reveal that Ppm1b negatively regulates 3-bromopyruvic acid induced necroptosis in MDA-MB-231 cells that correlates with enhanced dephosphorylation of RIP3. We found that 3BP was able to directly suppress its target Ppm1b, thereby impairing proliferation and inducing necroptosis in breast cancer cells. This mechanism involved in regulation of Ppm1b on necroptosis highlight the potential role of Ppm1b as a therapeutic target to treat breast cancers. Which part of the stage of the development of breast cancer cells does Ppm1b involved in is still clear, which needs to be investigated with further research.

## Data Availability Statement

The original contributions presented in the study are included in the article/**Supplementary Material**, further inquiries can be directed to the corresponding author.

## Ethics Statement

The animal study was reviewed and approved by Bengbu Medical College Institutional Animal Care and Use Committee.

## Author Contributions

YS and QP provided intellectual contributions in the design of the study, generated all the results in this study, and wrote the manuscript. SZ and HL reviewed the manuscript. LM and CC helped in tumor measurements in mice and contributed to the study design including reviewing the manuscript. YS, QP, and HL are the principal investigators who designed the study and wrote the main draft of the manuscript. All authors contributed to the article and approved the submitted version.

## Funding

Funding support for this work was provided by The National Science Foundation of China (81372899), The Provincial Science and Technology Cooperation Project of Anhui province (1503062024), The key University Natural Science Project of Anhui Province (KJ2016A486), The Natural Science Foundation of Anhui province (1508085MH166), and The Foundation of Bengbu Medical College (Byycxz1635, BYKY2019024ZD).

## Conflict of Interest

The authors declare that the research was conducted in the absence of any commercial or financial relationships that could be construed as a potential conflict of interest.

## Supplementary Material

Supplementary Video 1 Live-cell observation of MDA-MB-231 cells after incubation with 3-BP. Results shown that disruption of plasma membranes of MDA-MB-231 cells after incubation with 3-BP for 24 h and cell fragments are visible, resulting in the release of cell contents, swollen nuclei (N) and cytoplasmic material are visible, which mean that 3-BP may induce breast cancer cells MDA-MB-231 necroptosis.

Supplementary Video 2 Live-cell observation of MCF-7 cells after incubation 24h with 3-BP. Results shown that the characteristics of apoptotic cell death, with typical apoptotic bodies, and the number of apoptotic nuclei was significantly increased, which mean that 3-BP may induce breast cancer cells MCF-7 apoptosis.
